The article "Image Recognition of Sports Athletes' High-Intensity Sports Injuries Based on Binocular Stereo Vision" was retracted in 2023. Reasons: unreliable results or conclusions; concerns about the data; concerns about the results or conclusions; concerns about the peer review.

# Image Recognition of Sports Athletes' High-Intensity Sports Injuries Based on Binocular Stereo Vision

**DOI:** 10.1155/2022/4322597

**Published:** 2022-07-31

**Authors:** Dongdong Chen

**Affiliations:** Xinyang Normal University, Xinyang 464000, China

## Abstract

Sports athletes are prone to certain injuries during high-intensity exercise training. In the process of treating an injury, images of the injury site need to be collected and identified. However, the traditional recognition method cannot effectively extract the features of the image. At the same time, it ignores the optimization of the damage image recognition results, resulting in low recognition accuracy and poor efficiency. Binocular stereo vision technology can quickly and accurately detect moving objects. Therefore, in order to more accurately identify high-intensity sports injury images, this study takes the high-intensity sports injury images as the basic research object. Several processes of image processing based on binocular stereo vision are analyzed, and the vulnerable parts of the body in high-intensity sports are also studied. Finally, the method in this study is verified. The experimental results show that the method proposed in this study reduces the average error rate by 0.19% compared with the traditional recognition method. It can effectively identify and detect injury images, thereby improving the accuracy and stability of sports injury image identification. The  identification time is also shortened accordingly, which has certain practicability and feasibility. In addition, the binocular camera used in this study has high accuracy, and the obtained images of sports injuries are of good quality, which lays a foundation for image detection and recognition.

## 1. Introduction

Athletes who participate in high-intensity and technically difficult sports are more likely to sustain injuries during exercise, such as cervical spine and lumbar spine injuries. Binocular stereo vision closely resembles how the human eye processes images. It is a very dependable and simple algorithm that has proven its worth in a variety of fields. As a result, this study proposes a binocular stereo vision-based recognition method for high-intensity sports injury images, which is critical for the repair and treatment of injured athletes' parts.

Timely detection and identification of injury sites in athletes can more accurately diagnose the type and severity of injuries. Some scholars have conducted some studies on the identification of sports injuries. Prabhu et al. discovered that diffusion tensor imaging, magnetic resonance spectroscopy, and fMRI can detect changes in encephalopathy. The pathological examinations he performed documented progressive neuronal degeneration of the tau protein. It was found that prevention, early diagnosis, and appropriate treatment are the recommended methods for the treatment of these diseases [1]. Zhu et al. used a research method based on big data technology and CNN-based computer vision technology and theoretical analysis related to sports mechanics and image recognition. His research provided technical support for injury risk prediction in athletes [2]. Wang research purpose is to find how to intelligently process images of soccer games based on computer intelligence techniques. First of all, he identified and processed the dynamic images of sports and collected static and dynamic images of football. The experimental results showed that the systematic error of the auxiliary identification technology based on the Internet of things is 0.63. So, his proposed algorithm and the obtained experimental results effectively demonstrate the reliability of using intelligent image recognition techniques for soccer sports image recognition [3]. Based on the characteristics of athletes, Ma et al. developed and designed a C/S mode athlete training process monitoring system, using GPS to obtain real-time position information of athletes. In order to reveal the changing laws of various indicators of athletes under training, he followed a series of physical conditions of the athletes, such as the characteristics of physical functions, training programs and arrangements, the status of brain functions, routine physiological and biochemical indicators, and basic conditions of injuries [4]. The above researchers have combined the treatment and prediction of sports injuries with intelligent technology, which has played a certain role in promoting the recovery of athletes, but they did not put it into practice and lacked reliability.

Binocular stereo vision technology is a high-speed, high-precision noncontact measurement method. For this technology, many scholars have conducted research. Lin et al. aimed to develop a 3D image reconstruction method based on laser line scanning (LLS) technology to establish a binocular stereo vision system for preliminary research on obstacle detection technology for autonomous underwater vehicles (AUVs). Therefore, the results of the stereo vision system evaluation demonstrate the reliability and performance of the tank [5]. Based on the binocular stereo vision measurement principle and wireless sensing theory, Li and Zhang studied the measurement and analysis method of the athlete's movement displacement parameters. He developed a noncontact displacement measurement system. The experimental results showed that the integrated displacement measurement system designed in this study has high precision and good stability [6]. Lin et al. discussed one of the foundations of 3D reconstruction methods in binocular stereo vision, that is, feature matching. He studied the operation principles, feature matching algorithms of binocular stereo vision system, and 3D reconstruction system. Based on these studies, he proposed a set of more feasible algorithms to improve the effect of 3D reconstruction [7]. Sun et al. established a perspective projection model of any section of the elbow. Based on this model, he proposed a method to locate the precise projected position of the on-axis point on the image plane and reconstruct the 3D coordinates of the on-axis point using binocular stereo vision. He measured three bends of different diameters. Compared with the classical method, this method effectively reduced the reconstruction error [8]. The abovementioned scholars used this technology to analyze their research objects and proved the reliability and stability of this technology, but they did not conduct experiments on its application and lacked data support.

After a series of experimental analysis, it can be concluded that the error of the method in this study for the coordinate positioning of the damage image is less than 0.5 mm, and the error rate is less than 2%. This shows that the method in this study can locate the damage target more accurately. The recognition rate of the method in this study is significantly higher than that of other methods, and the lowest is more than 60%, which proves the operability of the method. In addition, the method proposed in this study consumes the shortest time when the number of recognized images is different, and the lowest is 0.5 seconds. This also shows that the recognition rate of this method is the highest, and it has great advantages over other methods. As the number of experiments increases, the error rates of different methods show different trends. The error rate of the method proposed in this study is much lower than other methods, with an average of about 0.06%, and that of other methods is about 0.25%. This shows that the method proposed in this study can reduce the error to a relatively low level when recognizing sports-impaired images.

## 2. Binocular Stereo Vision, High-Intensity Sports Injury, and Image Recognition

### 2.1. Binocular Stereo Vision

There are many ways that humans get information, and 70 percent of it comes from what people see. Therefore, vision has played an extremely important role in the process of people observing the world and understanding the world. Studies have shown that when people see things with the left eye and see things with the right eye, their perception of distance and spatial perception of objects will become different. The reason for this phenomenon is that the positions of the two eyes of human beings are different, which makes the things and images seen by the left eye and the right eye different. However, when the left and right eyes look at things at the same time, the neural tissue of the brain will fuse the received image information to form a sense of space for the object. This formation process is called binocular stereo vision. It is generally called BSV, that is, binocular stereo vision. Binocular stereo vision is an important part of computer vision [9–11].

The theoretical basis of binocular stereo vision technology is parallax theory (as long as the parallax angle and the baseline length are known, the distance between the target and the observer can be calculated). The main purpose of this technology is to restore and reconstruct the depth information and three-dimensional geometric coordinates of pixels, the purpose of which is mainly achieved by acquiring images. The “image” here is based on the simultaneous acquisition of the left and right perspectives, so it has certain passivity. With this technology, the real three-dimensional world can be quickly restored, providing the user with a description of the location of the target during the navigation process. Binocular stereo vision technology is more comprehensive, and it contains a variety of subject knowledge, such as optics, physics, and computer science. The most difficult and critical component of binocular stereo vision technology is the process of camera position calibration and feature matching. The model structure based on binocular stereo vision is extremely simple, and the operation efficiency is also very high, so its application prospect is very broad. In particular, this model is widely used in the automated production of factories. The human eye is capable of perceiving three-dimensional objects in three dimensions, and binocular stereo vision systems mimic this criterion. The simulation process is based on the principle of triangulation. This system uses imaging equipment and a computer to perform a series of processing on images. The system is generally divided into four functional modules, as shown in Figure 1.

Next, the binocular stereo vision system will be introduced in detail. It consists of three components, namely a binocular camera, a frame grabber, and a computer. First, as the name implies, the binocular camera has two cameras, which also allows it to collect two images of the detected object from different positions. Second, the image acquisition card is connected to the camera and the computer, and the specific process is as follows: first, the binocular camera collects the image signal. Then, the acquisition card converts the collected signal into a digital signal and then transmits the digital signal to the computer. The computer saves it to the hard disk. Third, the computer mainly completes a series of tasks through algorithms, including image preprocessing and segmentation, feature extraction, and stereo matching, to calculate the three-dimensional geometric information of the detected graphics and reconstruct the three-dimensional scene. The basic principle of binocular stereo vision is shown in Figure 2.

The image processing process of binocular stereo vision will be introduced in detail as follows:

1. *Image Preprocessing* [12, 13]. The camera can capture the image of the detected object, and then, the capture card transmits the image captured by the camera to the computer. In this process, it is easy to be subject to various interferences, which leads to the degradation of image quality and brings certain difficulties to subsequent image recognition. Therefore, image preprocessing becomes a necessity. The main purpose of image preprocessing is to remove the interference factors in the transmission process and enhance the pixels of the detected object in the image. If this task is done well, it will be more conducive to feature extraction and stereo matching of detected objects. In addition, this process can operate in both spatial (the two-dimensional plane where the image plane is located) and frequency (the spatial frequency of the gray value of the image pixel changing with the position) domains simultaneously, so it can also effectively reduce noise.
2. *Selection of Color Space*. When processing more complex images, people usually select the part they are interested in and extract the feature information of this part. This process is called image processing. The basic flow of general image processing and recognition is shown in Figure 3. The result frame of image recognition based on binocular stereo vision is shown in Figure 4. For image information of different difficulties, it is necessary to select an appropriate color model, so as to facilitate its analysis, and also help computer equipment to quickly identify the characteristic information of the image. There are many general color models. Among them, hue, saturation, and intensity (HSI), luminance a and b (Lab), cyan, magenta, and yellow (CMY), red, green, and blue (RGB) are relatively common, which have different characteristics.
3. *Image Segmentation*. Image segmentation [14, 15] refers to dividing the basic information of an image into several parts according to different characteristics. These parts are called image elements. The advantage of doing this is that it is conducive to fast matching of features. Each image element has its own characteristics, so they are also very easy to identify and distinguish. The advantage of image segmentation is that it can greatly reduce the workload of computers and administrators, thereby further improving the recognition efficiency of computers [16]. In general, there are various methods and classification criteria for image segmentation, mainly because the basis of segmentation is different. Among them, there are mainly three segmentation methods based on gray threshold, region growth, and edge detection. Among them, the first method is further divided into the maximum value method, the average method, and the weighted average method, as shown in Table 1.
4. *Extraction of Image Features*. What this process needs to do is to compare the different features of the two images, so that the coordinates of the same point in the three-dimensional space in the two different images can be obtained. The features of images can be divided into local features (points, lines, surfaces) and global features (polygons, images) according to different classification [17] criteria, which can also be divided into color, texture, shape, spatial relationship features, etc. Different features use different algorithms.
5. *Stereo Matching Process*. Stereo relative refers to two images taken by two cameras in a binocular camera of the same object. The purpose of stereo matching is to discover and find the coordinates and relationships of the corresponding points in the two images, which is also the focus of 3D reconstruction. Stereo matching is also known as disparity estimation, or binocular depth estimation. Two algorithms are available for this process, that is, local descriptions based on invariants and statistical learning methods. This process is unique and reproducible, with some physical meaning.

### 2.2. High-Intensity Sports Injuries

High-intensity exercise training can greatly enhance the function of the human body, so that the maximum oxygen uptake of the organism can be improved, and myocardial functions such as heart rate, speed, and endurance can be improved [18]. The main characteristics of high-intensity exercise training are shown in Table 2. Under normal circumstances, the main contents of high-intensity exercise training include running and leapfrog, as shown in Table 3.

Sports injuries are clinically manifested as pain, swelling, etc., at the injury site of different severities. High exercise intensity is more likely to lead to muscle damage. As the name suggests, sports injuries refer to various injuries suffered by athletes during sports training [19]. Sports injuries are closely related to a series of factors, such as the intensity of sports, the type of sports, training environment, and sports auxiliary equipment. The specific classification of sports injuries is shown in Table 4.

In real life, injuries to athletes are unavoidable because most high-intensity sports involve relatively intense confrontation. With the passage of time, the injury develops concealment and long-term characteristics, causing permanent damage to the athlete's body. Abrasions, sprains, strains, and joint injuries are all common types of injuries [20]. Abrasions are common in sports with more physical contact. Scratches can occur as a result of falls caused by low friction on the ground or excessive slippage, or as a result of collisions or scratched fingernails as a result of physical contact between athletes. Second, some high-intensity sports have an excessive range of motion, resulting in injuries to the athletes' soft tissues and ligaments, particularly in the ankle, knee, and waist joints. Third, one of the most common causes of injury is athletes' lack of warm-up and preparation. If the preparation is insufficient, the muscles, including the thighs, calves, shoulders, and backs, will not stretch. Fourth, if a joint injury, such as the metacarpophalangeal joints, ankle joints, or knee joints, persists, it is likely to become an old injury. Joint injuries are difficult to treat and can lead to complications.

According to the above analysis, the reasons for the injury can be summed up in three points, namely psychological reasons, physical quality, and objective factors. There are also some preventive measures and strategies for these three points, as shown in Table 5.

### 2.3. Image Recognition and Processing of High-Intensity Sports Injuries

To identify the injury image, the main cause of sports injury must first be determined. The formula for calculating the injury rate of each sport in high-intensity training is as follows:

(1) $$\begin{array}{c} \Delta \Delta \Delta E_{ℬ}\left(Y\right)=\frac{\sum_{i=1}^{\Delta }C_{\Delta \Delta \Delta }\left(\Delta_{\Delta \Delta }\right)}{ℒ\times \beta_{\Delta }}. \end{array}$$

In formula (1), *β*_Δ_ refers to the parts of the body that are easily damaged during high-intensity training; ℒ refers to the maximum heart rate before high-intensity exercise; and Δ_ΔΔ_ refers to the severity of the injury. *𝒞*_ΔΔΔ_ refers to different sports, and Δ refers to the number of vulnerable parts.

All factors that contribute to an athlete injury are as follows:

(2) $$\begin{array}{c} S=\frac{E_{\Delta }\left(Y\right)\cdot ℛ{}^{\prime }}{\Delta \times Y_{\ell \Delta \Delta }\cdot \Delta_{\Delta }}\cdot {ℬ}_{\ell \Delta \Delta }. \end{array}$$

In formula (2), ℬ_*ℓ*ΔΔ_ refers to the various causes of damage; *𝒴*_*ℓ*ΔΔ_ refers to the probability of various damage types; and *ℰ*_Δ_(*𝒴*) refers to the law of damage.

The relationship between high-intensity exercise training intensity and injury is as follows:

(3) $$\begin{array}{c} K_{\alpha }=\frac{\Delta \Delta \Delta G_{ℬ}\left(Y\right)}{S\times {ℬ}_{\ell \Delta \Delta }}\Delta S_{0}. \end{array}$$

In formula (3), *𝒮*_0_ refers to the probability of injury to various joint parts of sports players.

The relationship between sport and injury severity is as follows:

(4) $$\begin{array}{c} P_{\left(\Delta \right)}=\frac{\Delta_{\Delta }\cdot \Delta_{\Delta }\phi \left(\Delta_{\Delta }\right)}{\beta_{\Delta }}\times \frac{ℒ\left(\Delta ,\Delta_{\Delta }\right)}{\Delta_{\Delta \Delta }}+\Delta . \end{array}$$

In formula (4), Δ_Δ_ refers to the injury site; *ϕ* refers to the general pattern of the injury; and Δ_Δ_ refers to the duration of the sportsman's exercise. Δ refers to the important part of the injury. ℒ(Δ, Δ_Δ_) refers to the proportion of the number of people injured in each sport.

The statistical formula of the injured parts that sports athletes are prone to produce in the process of high-intensity sports training is as follows:

(5) $$\begin{array}{c} X_{\Delta }^{ℳ}=\frac{\left[\Delta_{\ell }\left(\Delta_{\Delta }\right)\cdot \Delta_{\Delta }\left(\Delta_{\Delta }\right)\right]}{{ℛ}_{s\Delta \Delta \Delta \Delta }\cdot {ℛ}_{\Delta \Delta \Delta }}\cdot \frac{\phi }{P_{\left(\Delta \right)}}. \end{array}$$

In formula (5), Δ refers to the cumulative number of injuries in sports athletes. Δ_*ℓ*_(Δ_Δ_) refers to the type of cause that causes the injury, and Δ_Δ_(Δ_Δ_) refers to the ratio of various causes of injury. ℛ_*𝒮*ΔΔΔΔ_ refers to the joints that are susceptible to injury, and ℛ_ΔΔΔ_ refers to the joints with the highest proportion.

The main factors of sports athlete injury are as follows:

(6) $$\begin{array}{c} E\left(A\right)=X_{\Delta }\frac{AP_{\left(\Delta \right)}}{Q_{\Delta \Delta }}\times Y. \end{array}$$

In formula (6), *𝒴* refers to the detection of high-intensity exercise training intensity.

The basic law of the formation of the main factors is as follows:

(7) $$\begin{array}{c} N_{\omega }=\frac{\Delta \left(ℬ\right)\Delta \gamma }{\beta \times \omega \cdot \alpha }. \end{array}$$

Here, *γ* refers to the maximum speed and endurance of the athlete, and *β* refers to the characteristics of the injury. *ω* refers to the probability of an injury occurring, and *α* refers to the severity of the injury.

The main factors of the injury are classified, the formula of which is as follows:

(8) $$\begin{array}{c} \Delta \Delta \Delta Y_{\Delta }=\Delta_{\Delta }\Delta_{\Delta }\cdot \frac{\Delta \Delta -\Delta_{\Delta \ell }}{\left(\Delta \left(\gamma \right)\mathrm{*\chi}\right)}\cdot \alpha N_{\varphi }. \end{array}$$

In formula (8), Δ(*γ*) refers to the variability of injuries among sports players, and *α* refers to the type and severity of injuries. Δ_Δ_Δ_Δ_ refers to the injury probability of each part; Δ_Δ*ℓ*_ refers to the probability of injury caused by strains and sprains; and *χ* refers to the training volume of athletes.

Then, the sports injuries and their causes are classified and counted. The formula is as follows:

(9) $$\begin{array}{c} U_{\Delta \Delta }\left(\Delta +1\right)=\frac{VU_{\Delta \Delta }+{ℬ}_{\Delta }\Delta_{\Delta \Delta }\left(\Delta \right)-Y_{\Delta \Delta }\left(\Delta \right)}{Y_{\Delta \Delta }\left(\Delta \right)+ℶ\cdot \Delta_{\Delta }}\Delta \Delta \Delta_{Y_{\Delta }}. \end{array}$$

In formula (9), ℶ refers to training phases with different intensities; Δ_Δ_ refers to training time; and *𝒰*_ΔΔ_ refers to the speed of the athlete. *𝒴*_ΔΔ_ refers to the endurance time of athletes; ℬ_Δ_ refers to the weight of the cause of injury; and Δ_ΔΔ_ refers to the injury rate caused by the characteristics of different sports. (Δ) refers to the training level of the athlete.

The relationship between the training history process and the probability of sports injury is expressed as follows:

(10) $$\begin{array}{c} G=\frac{\theta }{\Delta_{\Delta }\Delta \cdot \delta }P*U_{\Delta \Delta }\left(\Delta +1\right). \end{array}$$

In formula (10), *θ* refers to the historical process of an athlete's injury; Δ_Δ_ refers to the injury samples collected; and *𝒫* refers to the basic situation and data information of the athlete.

After analyzing the cause of the injury, the grayscale conversion operation on the image of sports injury can be performed. If the motion-impaired image is colored, its pixels are represented by three bytes, which correspond to the brightness generated by the three components of R, G, and B. The formula for grayscale conversion is as follows:

(11) $$\begin{array}{c} G\Delta \Delta \Delta \left(\Delta ,\Delta \right)=S\left(\Delta ,\Delta \right)+ℱ\left(\Delta ,\Delta \right)+A\left(\Delta ,\Delta \right). \end{array}$$

The converted grayscale image is represented by a 24-bit image, which can effectively improve the recognition efficiency of high-intensity sports injury images. To further improve the recognition effect of sports injury images, it is necessary to extract the basic contour of the injury site. According to the characteristics of the damage image itself, the curve fitting method (substituting the existing data into a mathematical expression through mathematical methods) is used to obtain the final damage contour.

To make the model of the damaged contour reach a state where the active contour converges on the edge of the damaged part, the contour energy is calculated. Its formula is as follows:

(12) $$\begin{array}{c} ℱ\left(ℬ\right)=\left[\beta {ℱ}_{\Delta \Delta }\left(ℬ\right)+\alpha {ℱ}_{\Delta \Delta }\left(ℬ\right)\right]G\Delta \Delta \Delta \left(\Delta ,\Delta \right). \end{array}$$

Here, ℱ(ℬ) refers to the energy value of the broken contour, and ℱ_ΔΔ_(ℬ) refers to the internal energy value of the active contour. ℱ_ΔΔ_(ℬ) refers to the external energy value of the active contour. *β* and *α* refer to the weight coefficient.

The image is divided to get the center of the target contour. The formula is as follows:

(13) $$\begin{array}{c} \bar{\Delta }=\frac{1}{\Delta }\sum_{\Delta =1}^{\Delta }\Delta_{\Delta }, \end{array}$$

(14) $$\begin{array}{c} \bar{\Delta }=\frac{1}{\Delta }\overset{\Delta }{\underset{\Delta =1}{\sum }}\Delta_{\Delta }. \end{array}$$

After the basic contour of the damage is extracted, the transformation analysis method is used to initially identify the damage site. The digital matrix is constructed according to the obtained number and information of the pixel points of the damaged position. To improve the recognition accuracy, the length pattern with the feature vector of sixty-four is selected. The mean of the image population vector is as follows:

(15) $$\begin{array}{c} \lambda =\frac{1}{\Delta }\sum_{\Delta =1}^{\Delta }\Delta_{\Delta }\cdot ℱ\left(ℬ\right). \end{array}$$

In formula (15), Δ refers to the number of sports injury images.

Next, a matrix ℬ is set and the eigenvectors of the covariance matrix are calculated. The formula is as follows:

(16) $$\begin{array}{c} \Delta_{\Delta }=ℬ\frac{1}{\sqrt{\mu_{\Delta }}}Y\cdot \Delta_{\Delta }\cdot \mathrm{\lambda .} \end{array}$$

Here, Δ_Δ_ refers to the eigenvector values of the matrix and *μ*_Δ_ refers to the nonzero eigenvalues of the matrix. Δ_Δ_ refers to the vector corresponding to the nonzero eigenvalues.

All training samples and image samples are projected into eigenspace *𝒯*, and the projection coefficient is calculated. The formula is as follows:

(17) $$\begin{array}{c} \Delta_{\Delta }=T^{S}\cdot \Delta_{\Delta }. \end{array}$$

Next, the Euclidean distance is used to calculate the minimum distance, which is the initial recognition result of the image sample. The calculation formula is as follows:

(18) $$\begin{array}{c} \Delta \left(\Delta ,\Delta \right)={\left[\overset{\Delta }{\underset{\Delta =1}{\sum }}{\left(\Delta_{\Delta }-\Delta_{\Delta }\right)}^{2}\right]}^{1/2}. \end{array}$$

Here, Δ(Δ, Δ) refers to the Euclidean distance (the straight-line distance between two points in Euclidean space) between image samples and training samples, and Δ refers to the number of training samples.

Next, the binocular stereo vision algorithm is used to further identify it, and the area of the damaged part is calculated. Then, the function of the position target of the camera can be expressed as follows:

(19) $$\begin{array}{c} K_{\Delta }=\sum_{\Delta =1}^{\Delta }U_{\Delta }-\Delta_{\Delta }^{2}\cdot \Delta \left(\Delta ,\Delta \right). \end{array}$$

Here, *𝒰*_Δ_ refers to the pixel cluster center, and Δ refers to the number of pixel cluster centers of the camera. Δ_Δ_ refers to the clustered object, and the minimum value of *𝒦*_Δ_ is the best clustering point, that is, ΔΔΔ_*𝒦*_Δ__.

Combined with the above analysis, the relative area of the damage image can be calculated, namely as follows:

(20) $$\begin{array}{c} A\Delta \Delta \Delta_{\ell \Delta \Delta \Delta \Delta }=\left(\frac{V{}^{\prime }}{C{}^{\prime }}\right)\cdot \left(\frac{G{}^{\prime }}{C{}^{\prime }}\right). \end{array}$$

Here, *𝒱*^*∗*^ refers to the number of long pixels in the lesion image; *𝒢*^*∗*^ refers to the number of wide pixels in the lesion image; and *𝒞*^*∗*^ refers to the resolution of the image.

After segmenting the image, the absolute area of the damaged image is as follows:

(21) $$\begin{array}{c} A\Delta \Delta \Delta_{\Delta }=\frac{Q}{Q{}^{\prime }}\cdot A\Delta \Delta \Delta_{\Delta \Delta \Delta \Delta \ell }\cdot \Delta \Delta \Delta_{K_{\Delta }}. \end{array}$$

Here, *𝒜*ΔΔΔ_Δ_ refers to the pixel area of the damaged part; 𝒬 refers to the total number of pixels in the damaged part; and 𝒬^*∗*^ refers to the total number of image pixels.

## 3. Comparison of Recognition Effects of Different Damage Detection Methods

To identify images of sports injuries, it is first necessary to locate the injury target. Next, some samples of sports injury images are selected, and then, three-dimensional reconstruction is performed on the coordinates in the samples, to perform the localization test of the method proposed in this study. The result obtained is shown in Figure 5.

According to Figure 5, it can be known that the error between the method in this study and the actual value is less than 0.5 mm, and the error rate is less than 2%. This shows that the method in this study can locate the damage target more accurately. Next, to verify the overall performance of high-intensity sports injury image recognition based on binocular stereo vision proposed in this study, one hundred athletes are selected, whose specific conditions are shown in Table 6.

Then, the instrument of the binocular stereo vision system is used to collect the data of the injured part of the subject. It is compared with other injury detection methods, to verify the recognition efficiency and time-consuming of the method in this study. Other damage detection methods include linear discrimination, ultrasound image features, and improved spectral clustering. For the convenience of expression, these methods are abbreviated as linear discriminant (LD), UIF, and ISC, respectively.  Figure 6 shows the recognition rate results of different methods of damage detection.

It is obvious from the experimental data in Figure 6 that the recognition rate of the first two methods is an inverted U-shaped curve, and the recognition rate is relatively low as a whole. The recognition rate of the third method fluctuates greatly and is extremely unstable, so it is not very feasible. The recognition rate of the method in this study is significantly higher than other methods, and the lowest is more than 60%, which proves the operability of the method. In fact, the number of images to be recognized also has a certain impact on the recognition rate. Therefore, the selection of the detection method is adjusted, and the improved spectral clustering is replaced by the wavelet coefficient Hu; that is, the LD, UIF, WCHU, and the method in this study are compared. The results are shown in Figure 7.

According to the data in Figure 7, it can be seen that the method proposed in this study consumes the shortest time when the number of recognized images is different, with a minimum of 0.5 seconds. This also shows that the recognition rate of this method is the highest, and it has great advantages over other methods. Next, different times of experiments are carried out, and the recognition error rates of these methods are compared. The comparison results are shown in Figure 8.

According to the data in Figure 8, it can be seen that with the increase in the number of experiments, the error rates of different methods show different development trends. The error rate of the method proposed in this study is much lower than other methods, about 0.06% on average, and about 0.25% for other methods, which shows that the method proposed in this study can reduce the error to a relatively low level when recognizing images of sports injuries.

## 4. Conclusions

High-intensity sports injuries can take a variety of forms. The longer a training period lasts, the more likely an athlete's body part will sustain repeated injuries. As a result, current research is focusing on how to reduce sports-related injuries by identifying injury images. There have always been issues with low recognition precision and frequent occurrences of errors in the process of recognizing damage images. This study proposes a binocular stereo vision-based method for high-intensity sports injury image recognition, and the damaged images are processed, including contour extraction of damaged parts and pixel calculation. The experimental analysis demonstrates the method's reliability and applicability, which is embodied in high recognition accuracy, short recognition time, and high recognition performance. However, there are some drawbacks to the method proposed in this study. The recognition accuracy and speed of the method in this study need to be improved for images of damaged parts with less obvious edge features. In the future, more research into this area will be conducted.

## Figures and Tables

**Figure 1:** Functional modules of the binocular stereo vision system.

**Figure 2:** Basic principle of binocular stereo vision.

**Figure 3:** Basic flow chart of image recognition.

**Figure 4:** Structural framework of image recognition based on binocular stereo vision.

**Figure 5:** Comparison of 3D reconstruction coordinates and actual targets.

**Figure 6:** Comparison of recognition rates of different damage detection methods.

**Figure 7:** Time-consuming comparison of identification of different damage detection methods.

**Figure 8:** Comparison of error rates of different damage detection methods.

**Table 1:** Commonly used segmentation methods.

Segmentation method	Operation	Effect
Segmentation method based on gray threshold	Grayscale processing	Reduce redundant information
Segmentation method based on region growth	Split by pixel	Complete image extraction
Segmentation method based on edge detection	Split according to contour	Image segmentation

**Table 2:** Basic parameter information of high-intensity exercise training.

Items	Remarks
Environment	Aerobic environment
Maximum load intensity	75%–80%
Heart rate	About 140 times/min
Oxygen supply method	Intermittent load method

**Table 3:** Basic content of high-intensity exercise training.

Serial numbers	Contents	Exercise intensity
1	800 m jogging	6 min to complete
2	5 times × 5 m turn back to run	3 groups, rest 2 min between groups
3	50 m run	5 groups, rest 1 min between groups
4	Leapfrog	3 groups, each group 20 times, rest 3 min between groups
5	Squat	
6	Relax and stretch	5 min

**Table 4:** Basic classification of sports injuries.

Division angle	Classification	Remarks
Damage property	Chronic injury	Heavy local body load
	Acute injury	Muscle strain
Damaged tissue structure	Skin, muscle, joint, and nerve injury	
Damage degree	Mild injury	No effect on normal training or competition
	Moderate injury	Affect normal training or competition for over 1 day
	Severe injury	Need hospitalization

**Table 5:** Causes of sports injuries and their prevention strategies.

Reason	Specific description	Preventive measure
Psychological quality	Focus on tactical skills	Psychological counselling and mental health education
		Psychological supervision
	Less training	Soothe and regulate emotions
		Raise awareness of prevention

Physical quality	High physical consumption	Strengthen physical fitness and strength training
		Develop training programs
	High demand for strength	Improve basic physical fitness
		Standardize and correct tactical actions

Objective reasons	Improper infrastructure maintenance	Strict requirements and specifications
		Check the equipment regularly
	Clothing discomfort	Meet reasonable requirements
		Check and prevent damage

**Table 6:** Details of the experimental subjects.

Items	Remarks
Male/person	55
Female/person	45
Height range (cm)	162–183
Weight range (kg)	44–75
Training program	Weightlifting, long-distance running, long jump, high jump, basketball, football, table tennis

## Data Availability

The data used to support the findings of this study are available from the author upon request.
